The article "Effects of Buzhong Yiqi Decoction Combined with THP Bladder Perfusion on Postoperative Efficacy in Patients with Bladder Cancer" was published in 2021. Journal: Evid Based Complement Alternat Med.

# Effects of Buzhong Yiqi Decoction Combined with THP Bladder Perfusion on Postoperative Efficacy in Patients with Bladder Cancer

**DOI:** 10.1155/2021/3685213

**Published:** 2021-11-11

**Authors:** Yunfeng Wang, Yan Zhang, Zhongguo Liu, Qiuying Li, Huijing Jin

**Affiliations:** ^1^Department of Clinical Laboratory, Chengyang People's Hospital, Qingdao 266109, China; ^2^Department of Nutriology, Qingdao Hospital of Traditional Chinese Medicine, Qingdao Hiser Hospital, Qingdao 266033, China; ^3^Department of Urology Surgery, Qingdao Central Hospital, Qingdao University, Qingdao 266033, China; ^4^Department of Imaging, Zhangqiu District People's Hospital, Jinan 250200, China; ^5^Ward Department, Zhangqiu District People's Hospital, Jinan 250200, China

## Abstract

**Background:**

As a traditional Chinese medicine tonic, Buzhong Yiqi decoction has the effects of invigorating Qi and lifting Yang. In this study, the effects of Buzhong Yiqi Shenge decoction combined with THP bladder perfusion on postoperative efficacy in bladder cancer were investigated.

**Methods:**

A total of 70 cases of bladder cancer patients were divided into the experimental group and control group according to the random number table method, with 35 cases in each group. The control group was treated with THP bladder perfusion. The experimental group was treated with Buzhong Yiqi Shenge decoction on the basis of the control group. The number of urine white blood cells, VEGF level, the incidence of adverse reactions, and KPS score were compared between the two groups before and after treatment.

**Results:**

After 3 and 6 months of therapy, the KPS score of the experimental group increased significantly compared with the control group. However, after 12 months of treatment, there was no difference in KPS scores between the two groups. Moreover, there was no significant variation in serum VEGF between two groups after 3 months of treatment. However, Buzhong Yiqi decoction notably reduced the level of VEGF after 6 months and 12 months. After 3 months, the urine white blood cell count was lower in the experimental group than in the control group. After 6 and 12 months, there was no difference in urine white blood cell count between the two groups. Furthermore, a total of 14 patients in two groups had reoccurrence after one year. Our results showed that there was no significant difference in postoperative recurrence rate between the experimental group and the control group. The occurrence rates of frequent and urgent urination, nausea/loss, and abnormal urine routine of appetite in the experimental group were significantly lower than those in the control group. But there was no difference in the occurrence rate of low heat, hematuria between the experimental group and the control group.

**Conclusion:**

Buzhong Yiqi decoction combined with THP bladder perfusion has no advantage in the short-term recurrence rate of bladder cancer patients. However, Buzhong Yiqi decoction can alleviate the symptoms of adverse reactions and improve the quality of life of patients.

## 1. Introduction

Bladder cancer is a malignant tumor arising from bladder epithelium and stroma. Bladder cancer is a common tumor of the urinary system, and its morbidity and mortality rank at the forefront of malignant tumors [1]. According to clinical characteristics, bladder cancer can be divided into three types: nonmuscular invasive bladder cancer, muscular invasive bladder cancer, and metastatic bladder cancer [2]. Nonmuscular invasive bladder cancer is an early stage of bladder cancer, and transurethral resection of bladder tumor (TURBT) is the best therapeutic option [3]. However, patients are prone to recurrence after TURBT surgery, and the recurrence rate is as high as 70% [4]. Therefore, bladder perfusion of chemotherapy drugs is usually performed after TURBT surgery to prevent recurrence [5, 6]. The commonly used perfusion drugs are hydroxycamptothecin, theprubicin (THP), mitomycin, epirubicin, and BCG [7, 8]. However, a series of serious complications such as bladder contracture and chemical cystitis can be produced by routine perfusion therapy.

The etiology of bladder cancer is not well understood clinically so far, which may be associated with the internal and external factors. Intrinsic factors may have some genetic origin, while extrinsic factors may be related to the patient's eating habits, smoking, infectious diseases, and chemicals [9, 10]. Regarding pathogenesis and clinical signs, according to modern Chinese medicine approaches, generally the pathogenesis is a deficiency of Qi in the kidney and accumulation of dampness heat in the bladder [11]. Clinical observation data show that TCM has protective effects on the patients' circulatory system and digestive system [12]. Adding TCM to the chemotherapy can reduce the side effects of surgery and get better therapeutic effects [13–15]. Gong et al. reported that Qici Sanling decoction repressed cell growth by downregulating the Wnt/*β*-catenin pathway in bladder cancer [16]. Tanshinone IIA suppressed EEMT by inhibiting STAT3-CCL2 in bladder cancer [17]. Therefore, the clinical treatment of TCM combined with and Western medicine is a new way to improve the treatment of bladder cancer.

In this study, Buzhong Yiqi Shenge decoction combined with THP bladder instillation was used to treat nonmuscular invasive bladder cancer, and the postoperative recurrence rate and adverse reactions were observed. Our study could provide a potential clinical basis for the treatment of bladder cancer with integrated TCM and Western medicine.

## 2. Materials and Methods

### 2.1. General Information

Seventy patients with nonmuscular invasive bladder cancer who were treated at Chengyang People's Hospital, Qingdao, Shandong, China, between February 2019 and November 2020, were selected as the study subjects. There were 51 males and 19 females. The patients were 35–79 years old, with an average age of 58.9 ± 11.3 years. All patients were newly diagnosed with bladder cancer by biopsy and postoperative pathology. The diagnostic criteria were according to the Chinese Guidelines for the Diagnosis and Treatment of Urological Diseases in 2014. These patients were randomly divided into the control group and experimental group. The control group was treated with THP bladder perfusion. The experimental group received Buzhong Yiqi Shenge decoction on the basis of the control group. There was no statistical significance in age, gender, pathological grade, and clinical stage between the two groups (Table 1). All patients have signed the informed consent, and this study was approved by the Ethics Committee of the Chengyang People's Hospital, Qingdao, Shandong, China.

  Inclusion criteria: underwent TURBT surgery, diagnosed as nonmuscular invasive bladder cancer, the functions of the heart, lung, liver, and kidney were basically normal, and voluntarily participated in clinical studies and signed the informed consent.
  Exclusion criteria: with serious heart, liver, kidney, and other systemic diseases, allergic to the drug used in this study, pregnant or lactating women, and the observation period was less than 1 year.

### 2.2. Clinical Treatment

In the control group, TURBT surgery was performed, first with THP bladder perfusion within 24 hours after TURBT surgery. 30 mg THP (Shenzhen Main Luck Pharmaceuticals Inc., SFDA approval number: H10930105) was fully dissolved in 40 ml 5% glucose injection and injected into the bladder through a urethral catheter under aseptic condition. Perfusion was performed once a week for a total of 8 times and then once a month for a total of 10 times. THP bladder perfusion treatment lasted for one year.

The experimental group was treated with Buzhong Yiqi decoction on the basis of THP bladder perfusion in the control group. The prescription of Buzhong Yiqi decoction was as follows: 25 g Astragali Radix, 10 g Radix Ginseng, 10 g Radix Angelicae Gigantis, 6 g Radix Glycyrrhizae, 10 g Rhizoma Atractylodis, 10 g Rhizoma Cimicifugae, 10 g Pericarpium Aurantii Nobilis, and 10 g Radix Bupleuri. Usage: decocted in water, one dose a day, twice in the morning and evening on an empty stomach, until 1 year after surgery.

## 3. Observed Indicators

### 3.1. KPS Score

KPS score was based on the patient health status score in progress of clinical oncology. After 3, 6, and 12 months of treatment, patients in both groups were evaluated for KPS scores.

### 3.2. Serum VEGF Detection

After 3, 6, and 12 months, 5 ml of fasting peripheral venous blood was collected from the patients in the two groups. Serum was collected after centrifugation at 3000 r/min for 10 min. Serum VEGF levels were determined by the enzyme-linked immunosorbent assay (ELISA).

### 3.3. Routine Urine Cytology

Cytological examination of urine or bladder irrigated specimens is one of the main methods for diagnosing bladder cancer. The number of white blood cells in urine was counted by a urine microscopy.

### 3.4. The Recurrence Rates

Cystoscopy was performed once every after 6 months. If suspicious lesions were found, a pathological biopsy could be performed to determine whether the bladder cancer has recurred. Recurrence cases were recorded at 6 and 12 months after THP bladder perfusion.

### 3.5. Statistical Analysis

SPSS20.0 software was used for data analysis. The chi-square test was used for counting data analysis between the two groups, and the *t*-test was used for measurement data analysis. *P* < 0.05 was considered statistically significant.

## 4. Results

### 4.1. Comparison of KPS Scores between Two Groups

Sixty-five of the 70 patients completed the study. In the control group, 2 cases were lost during follow-up, and 1 case could not be reexamined on time. In the experimental group, 2 patients could not take Buzhong Yiqi decoction as prescribed. As given in Table 2, there was no difference in KPS scores between the two groups before treatment. After 3 and 6 months of treatment, the KPS score of the experimental group increased significantly compared with the control group. However, after 12 months of treatment, there was no difference in KPS scores between the two groups.

### 4.2. Comparison of Serum VEGF Level between Two Groups

Before treatment, there was no significant difference in serum VEGF between the two groups, and the same results were observed after 3 months of treatment. After 6 and 12 months of treatment, serum VEGF levels in the experimental group were significantly lower than those in the control group (Table 3). Therefore, Buzhong Yiqi decoction notably reduced the level of VEGF after 6 months and 12 months.

### 4.3. Comparison of Urine White Blood Cells between Two Groups

The urine white blood cell count of the two groups is given in Table 4. After 3 months, the urine white blood cell count was lower in the experimental group than in the control group. After 6 and 12 months, there was no difference in urine white blood cell count between the two groups (Table 4).

### 4.4. Comparison of Recurrence Rate between Two Groups

As given in Table 5, a total of 14 patients in two groups recurred after one year. In the control group, 6 patients of postoperative recurrence after half a year were found, with a recurrence rate of 18.75%. 8 patients with postoperative recurrence after one year were found in the control group, with a recurrence rate of 25.00%. In the experimental group, 4 patients had recurrence after half a year, with a recurrence rate of 12.12%, and 6 patients had recurrence after one year, with a recurrence rate of 18.18%. The results showed that there was no significant difference in postoperative recurrence rate between the experimental group and the control group. Therefore, Buzhong Yiqi decoction did not affect the recurrence of short-term bladder cancer patients.

### 4.5. Comparison of Adverse Reactions between Two Groups

Adverse reactions were observed in both groups during treatment. The occurrence rates of frequent and urgent urination, nausea/loss, and abnormal urine routine of appetite in the experimental group were significantly lower than those in the control group (Table 6). But there was no difference in the occurrence rate of low heat, hematuria between the experimental group and the control group (Table 6). Our results showed that Buzhong Yiqi decoction could effectively reduce the incidence of adverse reactions.

## 5. Discussion

Bladder perfusion is the main method to prevent postoperative recurrence of bladder cancer, which can prevent tumor invasion and effectively reduce recurrence [18]. Long-term bladder perfusion will inevitably lead to different degrees of adverse reactions in the body [19]. According to traditional medicine approaches, bladder cancer is mainly caused by deficiency of Qi in the kidney and accumulation of dampness, heat, and toxin in the bladder. TCM helps the body to recover vital Qi by strengthening the body and eliminating pathogenic factors, so as to improve the clinical symptoms, reduce toxic and side effects, and improve the quality of life of patients. For example, compound Fufang Fufangteng mixture can alleviate bladder irritation and gross hematuria caused by THP bladder perfusion and improve symptoms [20]. Liu et al. found that Xiaozheng decoction combined with hydroxycamptothecin can effectively reduce the incidence of adverse reactions and prevent postoperative recurrence of bladder cancer [21]. Furthermore, Zhibai Dihuang decoction combined cysteine injection therapy can prevent the toxic side effects and improve the amount of bioactive mass of bladder cancer with a syndrome of fire hyperactivity due to yin deficiency type [22]. Therefore, the combination of Chinese and Western medicine can improve clinical efficacy.

Our study showed that the adverse reactions in the treatment of the two groups were mainly manifested as nausea, loss of appetite, hematuria, frequent and urgent urination, abnormal urine routine, and low fever. Buzhong Yiqi decoction combined with THP bladder perfusion can reduce the incidence of nausea, loss of appetite, frequent and urgent urination, and abnormal urine routine and improve patients' quality of life. VEGF is highly specific and can induce the proliferation of vascular endothelial cells and promote the angiogenesis of tumor cells, which has a certain relationship with tumor recurrence. Therefore, detection of the VEGF level can be used to determine the status of tumor metastasis and treatment outcomes. In this study, it was found that Buzhong Yiqi decoction combined with THP bladder perfusion could reduce the serum VEGF level in postoperative patients with bladder cancer, which was beneficial to reduce tumor recurrence and metastasis. Moreover, the urine white blood cell count in the experimental group was significantly lower than that in the control group only after 3 months. The results showed that Buzhong Yiqi decoction could relieve short-term postoperative inflammatory reactions.

Buzhong Yiqi decoction is from the spleen and stomach theory written by Li Gao, a famous medical scientist in the Jin and Yuan Dynasties. The prescription has achieved good therapeutic outcomes in the internal medicine, surgery, gynecology, pediatrics, and other clinical departments. The therapeutic formula consists of eight herbs: Radix Astragali, Radix Ginseng, Radix Angelicae Gigantis, Radix Glycyrrhizae, Rhizoma Atractylodis, Rhizoma Cimicifugae, Pericarpium Aurantii Nobilis, and Radix Bupleuri. These herbs interact with each other to play the role of supplementing the middle and replenishing Qi, lifting Yang and lifting depression, warming, and removing heat. Modern studies have shown that Buzhong Yiqi decoction can regulate spleen and gastrointestinal function [23], immune function [24], antipyretic [7], and antitumor [25] and protect the myocardium [26].

## 6. Conclusion

In conclusion, Buzhong Yiqi decoction combined with THP bladder perfusion in the treatment of bladder cancer plays an essential role in reducing adverse reactions during chemotherapy. Buzhong Yiqi decoction combined with THP bladder perfusion in the treatment of bladder cancer has the potential for therapeutic application.

## Figures and Tables

**Table 1:** Comparison of general clinical data between two groups.

Clinical parameters	Experimental group (*n* = 35)	Control group (*n* = 35)	*X* ^2^	*P* value
Age (years)				
≤58	10	12	0.265	0.607
>58	25	23		
Gender				
Female	26	25	0.072	0.788
Male	9	10		
TNM stage				
Ta	26	23	0.612	0.434
T1	9	12		
Tumor grade				
G1	18	17	0.566	0.754
G2	14	13		
G3	3	5		

**Table 2:** Comparison of KPS scores between two groups.

	Before treatment	3 months after treatment	6 months after treatment	12 months after treatment
Control group	73.65 ± 4.61	78.15 ± 10.31	82.47 ± 6.26	88.61 ± 11.32
Experimental group	72.21 ± 6.34	83.54 ± 6.37	90.92 ± 9.38	92.23 ± 7.26
*t*	2.153	2.578	1.354	2.047
*P*	0.655	0.028	0.034	0.421

**Table 3:** Comparison of the serum VEGF level between two groups (pg/ml).

	Before treatment	3 months after treatment	6 months after treatment	12 months after treatment
Control group	379.1 ± 105.9	366.9 ± 120.1	353.7 ± 125.6	331.4 ± 135.2
Experimental group	381.4 ± 90.7	353.7 ± 110.4	329.5 ± 121.4	290.3 ± 142.8
*t*	0.914	2.563	1.685	2.264
*P*	0.745	0.306	0.042	0.027

**Table 4:** Comparison of urine white blood cells between two groups (cells/*μ*L).

	Before treatment	3 months after treatment	6 months after treatment	12 months after treatment
Control group	59.24 ± 6.41	25.26 ± 4.27	19.14 ± 2.41	9.37 ± 3.74
Experimental group	58.62 ± 8.36	20.14 ± 2.09	18.46 ± 3.12	9.10 ± 2.46
*t*	3.64	2.72	1.38	2.67
*P*	>0.05	0.037	>0.05	>0.05

**Table 5:** Comparison of recurrence rate between two groups.

	*n*	6 months after treatment		12 months after treatment	
		*n*	Recurrence rate (%)	*n*	Recurrence rate (%)
Control group	32	6	18.75	8	25.00
Experimental group	33	4	12.12	6	18.18
*X* ^*2*^			0.548		0.447
*P*			0.459		0.504

**Table 6:** Comparison of adverse reactions between two groups.

	*n*	Frequent and urgent urination	Nausea/loss of appetite	Low heat	Hematuria	Abnormal in urine routine
Control group	32	25 (78.13%)	16 (50.00%)	8 (25.00%)	11 (34.38%)	15 (46.88%)
Experimental group	33	12 (36.36%)	8 (24.24%)	5 (15.15%)	6 (18.18%)	7 (21.21%)
*X* ^*2*^		4.093	4.628	0.985	2.206	4.779
*P*		0.043	0.031	0.321	0.137	0.029

## Data Availability

The data used to support the findings of this study are available from the corresponding author upon request.

## References

[1] Bray F., Ferlay J., Soerjomataram I., Siegel R. L., Torre L. A., Jemal A. (2018). Global cancer statistics 2018: GLOBOCAN estimates of incidence and mortality worldwide for 36 cancers in 185 countries. *CA: A Cancer Journal for Clinicians*.

[2] Ferlay J., Soerjomataram I., Dikshit R. (2015). Cancer incidence and mortality worldwide: sources, methods and major patterns in GLOBOCAN 2012. *International Journal of Cancer*.

[3] Tran L., Xiao J.-F., Agarwal N., Duex J. E., Theodorescu D. (2021). Advances in bladder cancer biology and therapy. *Nature Reviews Cancer*.

[4] Zhai M., Tang C., Li M. (2020). Short-term mortality risks among patients with non-metastatic bladder cancer. *BMC Cancer*.

[5] Chen L., Hu W., Li G., Guo Y., Wan Z., Yu J. (2019). Efficacy of bladder perfusion of alternating hydroxycamptothecin and gemcitabine combined with low-dose tuberculin in the treatment of non-muscle invasive bladder cancer after TURBT. *Journal of B.U.ON: Official Journal of the Balkan Union of Oncology*.

[6] Taoka R., Tsunemori H., Matsuoka Y. (2021). Use of surgical checklist during transurethral resection increases detrusor muscle collection rate and improves recurrence‐free survival in patients with non‐muscle‐invasive bladder cancer. *International Journal of Urology*.

[7] Fujita N., Hatakeyama S., Momota M. (2020). Safety and efficacy of intensive instillation of low-dose pirarubicin vs. bacillus Calmette-Guérin in patients with high-risk non-muscle-invasive bladder cancer. *Urologic Oncology*.

[8] Wang T., Ding Y., Yang Y. (2019). Synergistic antitumour effects of triptolide plus 10-hydroxycamptothecin on bladder cancer. *Biomedicine & Pharmacotherapy*.

[9] Fang C. W., Hsieh V. C., Huang S. K., Tsai I. J., Muo C. H., Wu S. C. (2019). A population-based cohort study examining the association of documented bladder diverticulum and bladder cancer risk in urology patients. *PLoS One*.

[10] Adamowicz J., Juszczak K., Poletajew S., Van Breda S. V., Pokrywczynska M., Drewa T. (2019). Scented candles as an unrecognized factor that increases the risk of bladder cancer; is there enough evidence to raise a red flag?. *Cancer Prevention Research*.

[11] Zhou R., Hao L., Shi Z. (2018). Progress in TCM treatment of bladder cancer. *Journal of Clinical Medical*.

[12] Wang K., Chen Q., Shao Y. (2021). Anticancer activities of TCM and their active components against tumor metastasis. *Biomedicine & Pharmacotherapy*.

[13] Li T. F., Lin C. C., Tsai H. P., Hsu C. H., Fu S. L. (2014). Effects of Kuan-Sin-Yin decoction on immunomodulation and tumorigenesis in mouse tumor models. *BMC Complementary and Alternative Medicine*.

[14] Li C., Li M., Shu X. (2005). Toxicity attenuation and efficacy potentiation effects of sijunzi decoction on bladder carcinoma treated by chemotherapy in mice. *Chinese Journal of Integrated Traditional and Western Medicine*.

[15] Wang Y., Wang H., Zhang W. (2013). Genistein sensitizes bladder cancer cells to HCPT treatment in vitro and in vivo via ATM/NF-*κ*B/IKK pathway-induced apoptosis. *PLoS One*.

[16] Gong H., Chen W., Mi L. (2019). Qici Sanling decoction suppresses bladder cancer growth by inhibiting the Wnt/*β*-catenin pathway. *Pharmaceutical Biology*.

[17] Huang S. Y., Chang S. F., Liao K. F., Chiu S. C. (2017). Tanshinone IIA inhibits epithelial-mesenchymal transition in bladder cancer cells via modulation of STAT3-CCL2 signaling. *International Journal of Molecular Sciences*.

[18] Ba M., Cui S., Wang B. (2017). Bladder intracavitary hyperthermic perfusion chemotherapy for the prevention of recurrence of non-muscle invasive bladder cancer after transurethral resection. *Oncology Reports*.

[19] Sun K., Wang D., Wu G. (2021). Mirabegron improves the irritative symptoms caused by BCG immunotherapy after transurethral resection of bladder tumors. *Cancer medicine*.

[20] Zhou J., Gao H., Liang T., Liang X. (2016). Bladder perfusion THP combined oral compound fufang fufangteng mixture in bladder cancer TURBT postoperative clinical curative effect observation. *Chinese Journal of Cancer Prevention and Treatment*.

[21] Liu B., Yin X., Chen G., Bo H., Han B. (2018). Effect of Xiaozheng decoction combined with hydroxycamptothecin bladder instillation on postoperative recurrence of bladder tumor and serum VEGF. *Oncology Progress*.

[23] Peng Y., Jin J., Wu C., Yang J., Li X. (2008). Regulation of three Jianpi Buqi recipes on intestinal microflora of Piqi-deficiency rat. *China Journal of Chinese Materia Medica*.

[24] Utsuyama M., Seidlar H., Kitagawa M., Hirokawa K. (2001). Immunological restoration and anti-tumor effect by Japanese herbal medicine in aged mice. *Mechanisms of Ageing and Development*.

[25] Liu Y., Wang Y., Yi J., Jing H., Liu C. (2014). Effect of Buzhong Yiqi decoction on PI3K and AKT in spleen, stomach and lung of nude mice with lung adenocarcinoma transplantation tumor. *China Journal of Chinese Materia Medica*.

[26] Wang N., Zhang J., Xu H., Wang G., Chu L. (2011). Effects of buzhong yiqi decoction on adriamycin induced heart failure in rats. *China Journal of Chinese Materia Medica*.

